RETRACTED

# Inhibition airway remodeling and transforming growth factor-β1/Smad signaling pathway by astragalus extract in asthmatic mice

**DOI:** 10.3892/ijmm.2011.868

**Published:** 2011-12-23

**Authors:** ZHENG-HAI QU, ZHAO-CHUAN YANG, LEI CHEN, ZHI-DONG LV, MING-JI YI, NI RAN

**Affiliations:** 1 Department of Pediatrics, The Affiliated Hospital of Qingdao University Medical College, Qingdao 266003, P.R. China; 2 Department of Child Health Care, The Affiliated Hospital of Qingdao University Medical College, Qingdao 266003, P.R. China; 3 Department of Breast Surgery, The Affiliated Hospital of Qingdao University Medical College, Qingdao 266003, P.R. China

**Keywords:** astragalus plant, airway remodeling, asthma, trans-forming growth factor-β1/Smad signaling pathway

## Abstract

Airway remodeling is characterized by airway wall thickening, subepithelial fibrosis, increased smooth muscle mass, angiogenesis and increased mucous glands, which can lead to a chronic and obstinate asthma with pulmonary function depression. In the present study, we investigated whether the astragalus extract inhibits airway remodeling in a mouse asthma model and observed the effects of astragalus extract on the transforming growth factor-β1 (TGF-β1)/Smad signaling pathway in ovalbumin-sensitized mice. Mice were sensitized and challenged by ovalbumin to establish a model of asthma. Treatments included the astragalus extract and budesonide. Lung tissues were obtained for hematoxylin and eosin staining and Periodic acid-Schiff staining after the final ovalbumin challenge. Levels of TGF-β1 were assessed by immunohistology and ELISA, levels of TGF-β1 mRNA were measured by RT-PCR, and levels of P-Smad2/3 and T-Smad2/3 were assessed by western blotting. Astragalus extract and budesonide reduced allergen-induced increases in the thickness of bronchial airway and mucous gland hypertrophy, goblet cell hyperplasia and collagen deposition. Levels of lung TGF-β1, TGF-β1 mRNA and P-Smad2/3 were significantly reduced in mice treated with astragalus extract and budesonide. Astragalus extract improved asthma airway remodeling by inhibiting the expression of the TGF-β1/Smad signaling pathway, and may be a potential drug for the treatment of patients with a severe asthma airway.

## Introduction

The morbidity and mortality of asthma have increased sharply worldwide and it has become a severe global public health problem (1). The frequent occurrence of injury and repair initiated by chronic inflammation could lead to structural changes in the airway, collectively termed airway remodeling. Airway remodeling is characterized by airway wall thickening, subepithelial fibrosis, increased smooth muscle mass, angiogenesis and increased mucous glands (2,3). The direct consequence of the airway remodeling is persistent airway hyper-responsiveness and irreversible airway obstruction leading to a chronic and obstinate asthma with pulmonary function depression (4).

RETRACTED

*Astragalus membranaceus*, a is traditional chinese herbal medicine used for the treatment of the common cold, diarrhea, fatigue anorexia and cardiac diseases (5,6). It has also been used as an immunomodulating agent in treating immunodeficiency diseases and to alleviate the adverse effects of chemotherapeutic drugs. Research studies have been performed to investigate the usefulness of astragalus extract in the treatment of asthma, which can efficiently relieve symptoms and reduce the frequency of asthma attacks (7,8). However, little is known about the underlying mechanisms that regulate this activity.

Transforming growth factor-β1 (TGF-β1) is a pro-fibrotic cytokine thought to play an important role in promoting the structural changes of airway remodeling in asthma (9–11). Recently, the TGF-β1/Smad signaling pathway was found to be one of the important mechanisms involved in the development of airway remodeling in asthma (7,12,13). As important members of the TGF-β signal transduction system, Smad proteins directly transport signals from the cell membrane to the nucleus, and mediate intracellular TGF-β signal transduction regulating cell proliferation, transformation, synthesis, secretion and apoptosis. After being phosphorylated by the activated TGF-β1 receptor type I, Smad2 and Smad3 form a heterocomplex with co-Smad (Smad4), and transfer into the cellular nucleus activating DNA transcription to regulate the target gene expression. On the other hand, Smad6 and Smad7 can block the transcription induced by TGF-β through inhibiting its signaling pathway (14,15). Therefore, studies on signaling mechanisms, cytokines and their receptors in asthma could shed light on the mechanisms involved in airway remodeling and the treatment of asthma.

In this study, we report that astragalus extract inhibits airway remodeling in a mouse asthma model and regulates the TGF-β1/Smad signaling pathway in ovalbumin-sensitized mice, providing a novel mechanism for the astragalus extract inhibitory effect on airway remodeling in animal models of asthma.

## Materials and methods

### Reagents

Astragalus extract (formononetin and calycosin) were obtained from Haerbin Shengtai Botanical Development Co., Ltd. China; their chemical structures are shown in Fig. 1. Chicken egg ovalbumin (OVA) was purchased from Sigma (USA); TRIzol was purchased from Gibco-BRL (USA); the PCR kit was obtained from Promega (USA); the TGF-β1 ELISA-kit was purchased from R&D Systems (USA); Total Smad-2/3, phosphorylated-Smad2/3 antibodies, as well as secondary antibodies (P-Smad2 and P-Smad3) were purchased from Santa Cruz Biotechnology, Inc. (USA). Other laboratory reagents were obtained from Sigma.

RETRACTED

### Sensitization and antigen challenge

Forty-eight healthy female BABL/c mice, weighing 18–24 g were randomly divided into 4 groups, with 12 mice in each group: normal control group (A), asthma group (B), astragalus extract group (C), budesonide group (D). The asthmatic model were established by OVA. The mice were sensitized on Days 0, 7 and 14 by intraperitoneal injection of 20 μg OVA emulsified in 1 mg of aluminum hydroxide in a total volume of 0.2 ml in groups B, C and D. Seven days after the last sensitization, the mice were exposed to 1% OVA aerosol for up to 30 min every other day for 8 weeks. The 1% OVA aerosol was generated by a compressed air atomizer driven by filling a Perspex cylinder chamber (diameter 50 cm, height 50 cm) with a nebulized solution. Saline was used in group A instead of OVA. At the same time, mice in group C were treated with 0.4 ml (0.2 g/ml) astragalus extract by gavage before stimulation. Mice in group were treated with 4 ml (0.25 mg/ml) budesonide by atomization 15 min before stimulation and used as a drug control. All the experiments described below were performed in accordance with the regulations of the Centre of Animal Experiments of Qingdao University.

### Enzyme linked immunosorbent assay (ELISA)

At 24 h after the last challenge, bronchoalveolar lavage fluid was obtained from the mice under anaesthesia using 1 ml sterile isotonic saline. Lavage was performed four times in each mouse and the total volume was collected separately. The lavage fluid sample was immediately centrifuged at 2,000 rpm for 10 min at room temperature, and stored at -80°C until use. The TGF-β1 levels were then assayed with a TGF-β1 ELISA kit according to the manufacturer’s instructions. The data on the TGF-β1 protein levels were summarized as mean ± SE of each sample.

### Tissue samples

Lungs were removed from the mice after sacrificing 24 h after the last challenge. The tissues from the left lung were directly obtained from the surgical suite and immediately fixed in 10% buffered formalin and then embedded in paraffin. Sections (5 μm) were prepared and stained with hematoxylin and eosin (H&E). Additionally, Periodic acid-Schiff (PAS) staining was performed to identify mucus production in epithelial cells and the number of positive cells per unit length of basement membrane perimeter was determined. The thickness of the submesothelial extracellular matrix was determined after the tissue sections were H&E stained. The average of 10 independent measurements was calculated for each section and then the data were summarized.

RETRACTED

### Reverse transcription polymerase chain reaction (RT-PCR)

Total-RNA was isolated from the right lung tissue using the TRIzol reagent according to the manufacturer’s instructions. One microgram of the total cellular RNA was then reverse-transcribed into cDNA for PCR amplification using a kit from Sigma. The primer sequences used for PCR are listed in Table I. Amplification consisted of an initial 5 min incubation at 95°C and then 30 cycles of amplification using 30 sec of denaturation at 95°C, 30 sec at 57°C, and 60 sec at 72°C. The final extension was set for 10 min at 72°C. All data were expressed as the relative differences between control and treated cells after normalization to β-actin expression.

### Immunohistochemistry

The expression of TGF-β1 was assessed by semi-quantitative immunohistochemistry. After being deparaffinized, the sections were incubated in 0.01 mol/l citric acid buffer (pH 6.0) for 15 min in a microwave for antigen retrieval. After cooling, the sections were incubated in 3 g/l H_2_O_2_ for 30 min, to inactivate endogenous peroxidase. After blocking by 1:10 normal horse serum for 30 min, the supernatant was discarded. Primary anti-mouse TGF-β1 (1:300 dilution) was added overnight at 4°C. Then, biotinylated goat anti-rat secondary antibody and streptavidin horseradish peroxidase were added to the slides and incubated for 30 min at room temperature. Staining was completed by incubation with diaminobenzidine chromogen solution at room temperature. The stained cells were mounted and viewed under light microscopy.

### Westen blotting

Total protein was isolated from the right lung using a lysis buffer and quantified using protein quantification reagents from Bio-Rad. Next, 100 μg of the protein were suspended in 5X reducing sample buffer, boiled for 5 min, electrophoresed on 10% SDS-PAGE gels, and then transferred to polyvinylidene difluoride membranes by electroblotting. The membrane was blocked in 1% BSA/0.05% Tween-20/PBS solution overnight at 4°C, followed by incubation with the primary antibody for 24 h. A horseradish peroxidase-labeled IgG was used as the secondary antibody. The blots were then developed by incubation in a chemiluminescence substrate and exposed to X-ray films.

### Statistical analysis

Data are expressed as mean ± SD. Statistical comparisons of the data from the various groups were performed using the Student’s t-test. Differences between groups were considered statistically significant at P<0.05.

## Results

We have developed a mouse model of airway remodeling through repetitive OVA challenge. Mice were subjected to OVA challenge three times a week for 8 weeks and developed significant eosinophilic inflammation and airway remodeling similar to that observed in human chronic asthma.

RETRACTED

### Influence of astragalus extract on collagen deposition in asthma airway remodeling

We first stained and examined the histology of the airway wall in the four groups of mouse lung tissue. There was a little collagen deposition in the airway wall surrounding the normal mice, and the deposition increased significantly with an extensive distribution in the airway wall surrounding the asthma model mice (Fig. 2). Compared with the model group, collagen deposition in the mice treated with astragalus extract or budesonide was found to be significantly decreased (P<0.05).

### The effects of astragalus extract on goblet cell hyperplasia and mucus plugging of the airways

To identify the degree of goblet cells hyperplasia and mucus plugging of the airways, lung tissue sections obtained from mice 24 h after the last OVA challenge were stained with PAS staining. Compared to the control, goblet cells hyperplasia and mucus plugging in the OVA groups were significantly greater. However, the difference of goblet cells hyperplasia and mucus plugging between the astragalus extract and the budesonide groups was not significant (P>0.05) (Fig. 3).

### Effects of astragalus extract on TGF-β1 mRNA in mouse lung tissue

We next determined whether the astragalus extract can affect TGF-β1 mRNA production in the four groups of mouse lung tissue. Our data showed that, after an 8-week OVA-challenge, TGF-β1 mRNA expression in the OVA group was increased compared with the control group, whereas TGF-β1 mRNA expression in the astragalus extract and budesonide groups was decreased compared with that in the OVA group. There was no significant difference in TGF-β1 mRNA expressions among mice treated with astragalus extract and budesonide (P>0.05) (Fig. 4).

### Detection of TGF-β1 levels in the bronchoalveolar lavage fluid

We assayed TGF-β1 protein levels in the bronchoalveolar lavage fluid and found that TGF-β1 levels were significantly higher in asthmatic mice than those in the control group. Levels were even lower in washes from the astragalus extract-treated group and budesonide-treated group than in the asthmatic group (Fig. 5).

### Influence of astragalus extract on TGF-β1 expression in mouse lung tissue

TGF-β1 protein was found to be expressed in various cells of the lung including airway epithelial cells, fibroblasts, smooth muscle cells, vascular endothelial cells as well as the infiltrative inflammatory cells in model mice, while there was low expression of TGF-β1 protein in normal mice (Fig. 6). There was no significant difference in TGF-β1 expression in mice treated with astragalus extract and budesonide (P>0.05).

RETRACTED

### Effects of astragalus extract on Smad expression in mouse lung tissue

In order to investigate the expression of active TGF-β1 signaling *in situ*, we examined the expression of the intracellular effectors, Smads. An increase in the expression of P-Smad2/3 was observed during prolonged allergen challenge, whereas administration of astragalus extract and dexamethasone both considerably decreased P-Smad2/3 expression (Fig. 7). In contrast with P-Smad2/3, total Smad 2/3 (T-Smad2/3) expression levels remained unchanged. There was no significant difference of P-Smad2/3 in mice treated with astragalus extract and budesonide (P>0.05).

## Discussion

In the current study, we investigated the role of astragalus extract in the development of airway remodeling in asthma by immunohistochemistry and morphometric analysis of lung tissue *in vivo*. We identified an important role for astragalus extract in the progression of airway remodeling changes. Furthermore, we confirmed that the astragalus extract could modulate the expression of signaling molecules of the TGF-β1/Smad pathway, which may involved in modulating airway remodeling.

Airway remodeling is one of the pathophysiological characteristics of asthma, and its main pathological changes include subepithelial fibrosis formation and increased collagen deposition on the airway wall (16). Our study demonstrated the therapeutic effect of astragalus extract on airway remodeling in allergic airways disease. *Astragalus membranaceus* extract includes formononetin and calycosin, which have been identified as the major components responsible for the immunosuppressive and anti-inflammatory effects of this herb (17). The astragalus extract inhibits several pro-inflammatory cytokines and adhesion molecules that are important mediators of some autoimmune diseases, such as rheumatoid arthritis and asthma, and has been shown to be safe and clinically beneficial in these diseases (18). In the present study, we observed that the astragalus extract reduced collagen deposition and airway wall thickening involving the reticular basement membrane, smooth muscle layer and epithelial hyperplasia in the mouse model.

Steroids have been administered widely for their anti-proliferative activity in asthma airway remodeling, but they are not free of adverse effects (19). Such adverse reactions may be avoided if astragalus extract proves effective for the treatment of asthma airway remodeling. The present study indicated that astragalus extract could be a potential therapeutic agent for asthma by its anti-proliferative and anti-inflammatory properties. Compared with budesonide, they have equal ability to prevent asthma airway remodeling in our study. These findings further encourage the use of this small molecule in the treatment of asthma airway remodeling.

RETRACTED

How does the astragalus extract inhibit asthma airway remodeling? To use astragalus extract for clinical development effectively, it is essential to understand its mechanism. TGF-β1 is a potent fibrotic factor responsible for the synthesis of extracellular matrix. In recent years, a large number of studies demonstrated that TGF-β1 is an important cytokine in airway remodeling (20–22). Smads are the group of intracellular proteins that are critical for transmitting the TGF-β1 signals from the cell surface to the nucleus to promote transcription of target genes (23,24). In our study, we investigated the expression of active TGF-β1 signaling by detecting the expression of the intracellular effectors, Smads. Treatment with astragalus extract reduced the expression of TGF-β1 and TGF-β1 mRNA and modulated active TGF-β1 signaling in the airways, as demonstrated by a decrease in P-Smad2/3 expression. From our study, we can deduce that decrease of TGF-β1 levels and modulation of the activity of the TGF-β1 signaling pathway is a possible mechanism by which the astragalus extract inhibits airway remodeling in asthma.

In conclusion, our study demonstrated that the astragalus extract inhibited asthma airway wall remodeling through mechanisms involving a decrease in the production of TGF-β1 mRNA and TGF-β1 as well as modulation of active TGF-β1 signaling in the lung. It suggests the possibility of further developing astragalus extract as a candidate for the systemic therapy of asthma airway remodeling.

## Figures and Tables

**Figure 1:** Chemical structures of formononetin, calycosin.

**Figure 2:** Hematoxylin and eosin (H&E) staining of airway tissues in asthmatic mice. (A) Lung tissue sections obtained from mice 24 h after the last OVA challenge were stained with H&E, and all photos were captured at ×100 magnification. (a) Control group; (b) asthmatic group; (c) astragalus extract-treated group; (d) budesonide-treated group. (B) Morphometric parameters of airway tissues in four groups. Data are expressed as the mean ± standard error of the mean of at least 3 separate experiments.

**Figure 3:** Periodic acid-Schiff (PAS) staining of airway tissues in asthmatic mice. To identify the degree of goblet cells hyperplasia and mucus plugging of the airways, lung tissue sections obtained from mice on 24 h after the last OVA challenge were stained with PAS staining, and all photos were captured at ×100 magnification. (A) Control group; (B) asthmatic group; (C) astragalus extract-treated group; (D) budesonide-treated group.

RETRACTED

**Figure 4:** RT-PCR analysis of TGF-β1 mRNA in lung tissue. Mice were sacrificed 24 h after the final OVA challenge, and mRNA was then isolated and subjected to semi-quantitative RT-PCR analysis of TGF-β1. Expression of β-actin was used as a loading control. Lane M, marker; lane 1, control group; lane 2, asthmatic group; lane 3, astragalus extract-treated group; lane 4, budesonide-treated group.

**Figure 5:** ELISA analysis of TGF-β1 protein levels in bronchoalveolar lavage fluid. Bronchoalveolar lavage fluid was obtained from the mice under anaesthesia using 1 ml sterile isotonic saline and subjected to ELISA analysis. The data were summarized as mean ± standard error of the mean from at least 3 separate experiments. ^*^P<0.05 in comparison with the OVA group.

**Figure 6:** Effects of astragalus extract on the expression of TGF-β1 protein in the four groups of mouse lung tissue. Expression of TGF-β1 in lung tissue was determined by immunohistochemical staining. Positive staining is depicted in brown. Positive staining showed TGF-β1 expression in the epithelium, macrophage leukocytes and in smooth muscle. (A) Control group; (B) asthmatic group; (C) astragalus extract-treated group; (D) budesonide-treated group.

**Figure 7:** Effects of astragalus extract on Smad2 and 3 phosphorylation in lung tissue. Mice were sacrificed 24 h after the final OVA challenge. Total cellular protein was then extracted, and expression of P-Smad2/3 and T-Smad2/3 in lung tissue was determined by western blotting. Expression of GAPDH was used as a loading control.

**Table I:** Primers used for semi-quantitative RT-PCR.

Primer	Sequence	Length (bp)
TGF-β1-F	5′-GAAGTGGATCCACGAGCCCAAG-3′	247
TGF-β1-R	5′-GCTGCACTTGCAGGAGCGCAC-3′	
β-actin-F	5′-TTGATGTCACGCACGATTT-3′	222
β-actin-R	5′-GCTGTCCCTGTATGCCTCT-3′	
